# Additional baricitinib loading dose improves clinical outcome in COVID-19

**DOI:** 10.1515/med-2021-0010

**Published:** 2020-12-05

**Authors:** Md Jahidul Hasan, Raihan Rabbani, Ahmad Mursel Anam, Shihan Mahmud Redwanul Huq

**Affiliations:** Clinical Pharmacy Services, Department of Pharmacy, Square Hospitals Ltd, 18/F Bir Uttam Qazi Nuruzzaman Sarak, West Panthapath, Dhaka-1205, Bangladesh; Department of Medical Services, Internal Medicine and ICU, Square Hospitals Ltd, 18/F Bir Uttam Qazi Nuruzzaman Sarak, West Panthapath, Dhaka-1205, Bangladesh; Department of Medical Services, High Dependency Unit (HDU), Square Hospitals Ltd, 18/F Bir Uttam Qazi Nuruzzaman Sarak, West Panthapath, Dhaka-1205, Bangladesh

**Keywords:** baricitinib, COVID-19 pneumonia, loading dose, maintenance dose

## Abstract

Pneumonia associated with coronavirus disease 2019 (COVID-19) has been accounted for high mortality rate in severe COVID-19 worldwide, and additional serious scarcity of standard and effective anti-inflammatory drug in COVID-19 pneumonia management is a big challenge. Baricitinib, a Janus kinase (JAK) inhibitor, is a promising drug in COVID-19 pneumonia. This study aims to compare the clinical outcome of moderate-to-severe COVID-19 pneumonia treated with baricitinib with or without a loading dose. This prospective case-control study enrolled 37 adult patients where 17 patients (control) received baricitinib at 4 mg oral daily dose and 20 patients (case) received an additional single 8 mg oral loading dose. The median day to gain blood oxygen saturation level ≥95% (in room air) and return in normal breathing function were lower in case group than the control group. The requirement of intensive care unit and mechanical ventilation support was higher in the control group than in the case group [29.4% (*N* = 17)/10% (*N* = 20), *P* < 0.05; 11.8% (*N* = 17)/5% (*N* = 20), *P* > 0.05), respectively]. Thus, an additional loading dose of baricitinib revealed better clinical outcome of patients with COVID-19 pneumonia.

## 1 Introduction

The coronavirus disease 2019 (COVID-19) caused by severe acute respiratory syndrome coronavirus 2 (SARS-CoV-2), first introduces to the world as an outbreak in Wuhan, China, in December 2019, was declared as a “global pandemic” by World Health Organization (WHO) on March 11, 2020 [1]. As of July 11, 2020, a total of 12,322,395 confirmed COVID-19 cases and 5,56,335 related deaths have been reported worldwide [2]. Acute respiratory distress syndrome (ARDS) due to hyperinflammation in the lungs and ultimately, respiratory failure from COVID-19 pneumonia has been reported as the prime cause of COVID-19-associated mortality [3,4] ranging from 1% to more than 7% [5]. Cytokine storm due to the overproduction of proinflammatory cytokines, including interleukin (IL)-6, IL-7, IL-8, etc. in critically ill patients with COVID-19 is a critical phase of the disease that may lead to acute respiratory failure or multiple organ dysfunction [6,7]. Therefore, early detection of the COVID-19 infection and prompt management to suppress the cytokine storm is equally important in patients with COVID-19 [8].

IL-6 plays a pivotal role in exacerbating the cytokine storm as a part of host’s innate immune response mechanism that is mostly activated by IL-1 beta, tumor necrosis factor (TNF-alfa), Toll-like receptors (TLRs), prostaglandins, adipokines, and other cytokines [9]. High levels of IL-6 and IL-8 were detected in patients with severe SARS-CoV-1 infection, where high-magnitude of innate inflammatory response in correspondence to SARS-CoV-1 invasion in the host’s respiratory tract was extensively induced by IL-6 [10]. Similarly, high plasma level of IL-6 along with other proinflammatory cytokines, such as IL-2, IL-7, IL-8, IL-10, macrophage inflammatory protein (MIP1A), monocyte chemoattractant protein (MCP1), and TNF-alfa have been found in critically ill patients with COVID-19 and these cytokines significantly contribute in the severity of the disease [5,6,8].

Receptor-mediated endocytosis is a process through which most viruses penetrate the host cells. AP2-associated protein kinase 1 (AAK1) is a regulator of this endocytosis and inactivation of this enzyme interrupts the entry of the virus into the host cells [11]. Baricitinib, a janus kinase (JAK) inhibitor, is an approved drug for rheumatoid arthritis (RA). In effect, baricitinib specifically prevents the expression of proinflammatory cytokines, including IL-6 by inhibiting JAK. Interestingly, among the six highly potent inhibitors of AAK1, baricitinib is one of them which works by binding with the cyclin G-associated kinase that disrupts endocytosis, competently leading to a reduction in viral load [11,12]. Nowadays, baricitinib at a 4 mg once daily oral dose has been highlighted as a promising investigational anti-inflammatory (IL-6 inhibitor) drug therapy in patients with COVID-19 pneumonia [4,11,12,14]. The pharmacokinetics, pharmacodynamics, and safety data of baricitinib at a 4 mg daily dose in COVID-19 are still under investigation and to date, no standard dosing of baricitinib in COVID-19 has yet been established worldwide [11,12,13,14,15]. The objective of this study was to compare the clinical outcomes of patients with moderate-to-severe COVID-19 pneumonia treated with baricitinib at a 4 mg once daily oral dose with or without a high oral loading dose.

## 2 Materials and methods

### 2.1 Study design and data collection

This prospective case-control study was conducted in the “COVID-19 Unit” of Square Hospital Ltd, Dhaka, Bangladesh, on 37 adults (≥18 years) with moderate to severe COVID-19 symptoms admitted to this hospital from May 15 to June 13, 2020. All confirmed COVID-19 patients in this study were admitted to “COVID-19 unit” through a two-step triage system in the emergency department of the hospital. COVID-19 infection was confirmed in all patients by a positive reverse-transcriptase-polymerase-chain-reaction (RT-PCR) assay (instrument/device: Rotor Gene-Q/Cobas z480, and QIAGEN kits for real-time PCR, QIAGEN GmbH, Germany) of two specimens (nasal and oral swabs) in all patients collected by four trained phlebotomists following the hospital’s standard protocol of COVID-19 sample collection. All the patients were Bangladeshi citizens and older than 18 years. A combined dose of dexamethasone (corticosteroid) (10–20 mg/day, intravenously) and baricitinib was started on day 1 of admission for down-regulating the inflammatory processes in the lungs. Seventeen (*N*) patients in “no loading dose (LND) group” (control) received baricitinib 4 mg daily orally for 2 weeks, whereas 20 (*N*) patients in “loading dose (LD) group” (case) received baricitinib 8 mg single dose orally as a loading dose on day 1 and then 4 mg daily orally from days 2 to 14. The dose of baricitinib was taken on an empty stomach. Simple random sampling method was used in this study. The local brand “Baritor 2” (baricitinib 2 mg tablet) of Square Pharmaceuticals Ltd, Bangladesh, was used in this study. Data of this study were collected from online patient-wise data archive of this hospital and directly from patient-prescriptions on daily basis by participating doctors in COVID-19 unit. Adverse events were routinely monitored and reported by two clinical pharmacists.

The research related to human use has been complied with all the relevant national regulations, institutional policies, and in accordance with the tenets of the Declaration of Helsinki, and has been approved by the Research Ethics Committee, Square Hospitals Ltd, Dhaka, Bangladesh (no. 2004SH-OR024) on April 11, 2020. Written consent was taken from all participants in this study.

### 2.2 Inclusion criteria

Sample inclusion criteria were as follows:

(a) presence of SARS-CoV 2 in the nasal/oral swabs
(b) no previous history of COVID-19 infection
(c) having at least 3 of the following symptoms: fever, cough, tiredness, sore throat, anosmia, respiratory distress, and myalgia
(d) evidence of pneumonia in radiological diagnosis

### 2.3 Exclusion criteria

Sample exclusion criteria were as follows:

(a) more than 10 days from onset of symptoms
(b) patient with pregnancy
(c) any history of trauma or surgical procedure within the last 3 months of admission
(d) any history of acute/chronic autoimmune disease
(e) evidence of bacterial or fungal coinfection

### 2.4 Definition of moderate and severe COVID-19 pneumonia

Radiological evidence of bilateral pneumonia with clinical signs (fever, cough, difficulty breathing, tachypnea), no sign of severe stage of pneumonia, SpO_2_ (peripheral capillary blood oxygen saturation level) ≥90% on room air (RA), and ratio of arterial oxygen partial pressure to fractional inspired oxygen (PaO_2_/FiO_2_) 100–300 mmHg represents moderate COVID-19 pneumonia; radiological evidence of severe pneumonia with clinical signs (fever, cough, difficulty breathing, tachypnea) with at least one of the following signs: respiratory rate >30 breaths/min, severe respiratory distress, and SpO_2_ < 90% on room air represents severe COVID-19 pneumonia [16]. SpO_2_ ≥ 95% was considered as the targeted SpO_2_ in patients in this study. The severity of the disease and the progression of the symptoms of COVID-19 were measured on daily basis by assessing the physical condition of the patients and the laboratory investigations, including hematological tests, tests for liver and kidney functions, inflammation and infection markers, and arterial blood gas test.

### 2.5 Data analysis

Data were analyzed with SPSS version 22.0 statistical software (SPSS, Chicago, IL, USA). Descriptive statistics were presented through median value and interquartile range (IQR). Categorical variables were compared using Fisher’s exact test, and continuous variables were compared using Mann–Whitney *U* test. *P* values ≤ 0.05 were considered statistically significant.

## 3 Results

The number of male patients in both the groups was higher than the number of female patients with a median age of 52 (IQR: 50.5–62) and 59 (IQR: 49.8–69) in NLD and LD groups, respectively (*P* = 0.414). Fever [100 (IQR: 100–101.5)/100.5 (IQR: 100–101.75)], dry cough (100%, *n* = 17/100%, *n* = 20), generalized weakness (100%, *n* = 17/100%, *n* = 20), and sore throat (52.9%, *n* = 9/60%, *n* = 12) were significantly common in patients of NLD and LD groups (*N* = 17/20), respectively. Diabetes, hypertension, cardiovascular disease, bronchial asthma, chronic kidney disease, chronic obstructive pulmonary disease, obesity, malignancy, and Parkinson's disease were found as preexisting chronic diseases in patients with COVID-19 of NLD and LD groups (Table 1). Clinical characteristics, including blood-oxygen saturation profile, respiratory and cardiac functions, hematological components, and infection markers of all the patients in the two groups (NLD and LD) are given in Table 1 and compared, statistically.

**Table 1:** Baseline demographic, symptoms of COVID-19, comorbidity, and laboratory findings in patients treated with or without a loading dose of baricitinib

Characteristics	NLD group (control) (*N* = 17)	LD group (case) (*N* = 20)	*P* value
Male/female, *n* (%)	13/4 (76/24)	16/4 (80/20)	0.617
Age (year), median (IQR)	52 (50.5–62)	59 (49.8–69)	0.414
Days from onset of symptoms-to-hospitalization, median (IQR)	7 (4.5–7.5)	6.5 (5–7)	0.185
Fever (°F), median (IQR)	101 (100–101.5)	100.5 (100–101.75)	0.012
Dry cough, *n* (%)	17 (100)	20 (100)	0.001
Shortness of breath, *n* (%)	14 (82.4)	16 (80)	0.855
Weakness, *n* (%)	17 (100)	20 (100)	0.001
Diarrhea, *n* (%)	3 (17.6)	5 (25)	0.289
Anosmia, *n* (%)	11 (64.7)	14 (70)	0.516
Sore throat, *n* (%)	9 (52.9)	12 (60)	0.043
Diabetes, *n* (%)	14 (82.4)	17 (85)	0.675
Hypertension, *n* (%)	13 (76.5)	12 (60)	0.043
CVD, *n* (%)	6 (35.3)	4 (20)	0.052
Bronchial asthma, *n* (%)	4 (23.5)	6 (30)	0.389
CKD, *n* (%)	2 (11.8)	3 (15)	0.577
COPD, *n* (%)	2 (11.8)	3 (15)	0.577
Obesity, *n* (%)	2 (11.8)	2 (10)	0.740
Malignancy, *n* (%)	1 (5.9)	3 (15)	0.075
PD, *n* (%)	0 (0)	2 (10)	0.005
SpO_2_ (%), median (IQR)	89 (87.5–90)	89.5 (88–90)	0.718
Respiratory rate, (breaths/min), median (IQR)	22 (20.5–24)	23 (21–24)	0.825
PaO_2_/FiO_2_ (mmHg), median (IQR)	240 (195.5–263.5)	245 (193.8–262.3)	0.010
Heart rate (beat/min), median (IQR)	98 (85.5–105.5)	94.5 (84.5–113)	0.174
CRP (mg/L), median (IQR)	43.5 (30–220)	77.1 (40.9–211.5)	0.946
Procalcitonin (ng/mL), median (IQR)	0.12 (0.06–0.49)	0.18 (0.07–0.86)	0.062
WBC (K/µL), median (IQR)	6.3 (4.7–10)	8 (6.3–14.3)	0.021
Neutrophils (%), median (IQR)	87.6 (79.4–92.1)	82.5 (76.8–88.1)	0.657
Lymphocytes (%), median (IQR)	13.9 (11.9–15.8)	12.2 (8.2–14.5)	0.006
Platelet (K/µL), median (IQR)	186 (128–255)	175 (133.3–245.3)	0.605
d-Dimer (mg/L FEU), median (IQR)	2.7 (1.7–7.6)	2 (1.5–3.2)	0.018
Serum ferritin (ng/mL), median (IQR)	434 (293.5–543.5)	470 (361.3–604.8)	0.227
LDH ((U/L), median (IQR)	272 (216–404.5)	334 (295–390.5)	0.009
Creatinine (mg/dL), median (IQR)	0.9 (0.8–1)	0.9 (0.7–1.1)	0.210
ALT (U/L), median (IQR)	34 (29–57)	44 (35–54)	0.13
AST (U/L), median (IQR)	35 (25.5–49)	40 (29.5–58.8)	0.349
MEWS, median (IQR)	3 (2–3)	3 (2–3)	0.476

IQR = interquartile range; *n* = number; % = percentage; °F = grade Fahrenheit; CVD = cardiovascular disease; CKD = chronic kidney disease; COPD = chronic obstructive pulmonary disease; PD = Parkinson’s disease; SpO_2_ = peripheral capillary oxygen saturation; min = minute; PaO_2_/FiO_2_ = ratio of arterial oxygen partial pressure to fractional inspired oxygen; mmHg = millimetre of mercury; CRP = C-reactive protein; mg = milligram; L = liter; FEU = fibrinogen equivalent units; ng = nanogram; WBC = white blood cells; K/µL = thousand cells per micro liter; LDH = lactate dehydrogenase; U/L = units per liter; dL = deciliter; ALT = alanine aminotransferase; AST = aspartate aminotransferase; MEWS = Modified Early Warning Score.

All patients in both the groups tolerated baricitinib therapy well with no mild-to-serious adverse events (AEs) during the study period. No bacterial or fungal or any other opportunistic infections, hepatic or hematological toxicity were observed in the groups.

The median day to reach the targeted SpO_2_ (≥95% in RA) was less in the LD group (case) [3 (IQR: 2–8)] than that in the NLD group (control) [4 (IQR: 4–5)] (*P* = 0.180), and the median day to return in normal breathing function was significantly less in the LD group [5 (IQR: 4–5)] than that in the NLD group [8 (IQR: 7–10)]. ICU support was required higher in the NLD group with more requirement of mechanical ventilation support than that in the LD group [29.4% (*N* = 17)/10% (*N* = 20), *P* < 0.05; 11.8% (*N* = 17)/5% (*N* = 20), *P* = 0.141, respectively] (Table 2). The median day of hospitalization was lower in the LD group [12 (IQR: 10–14)] than that in the NLD group [15 (IQR: 9–18.5)] and this was statistically significant. The 30-day all-cause mortality rate was similar in NLD and LD groups [5.9%, *n* = 1 (*N* = 17)/5%, *n* = 1 (*N* = 20), respectively].

**Table 2:** Clinical outcomes in patients with COVID-19 treated with baricitinib with or without a loading dose

Parameters	NLD group (control) (*N* = 17)	LD group (case) (*N* = 20)	*P* value
Days required to increase SpO_2_ ≥ 95% in RA, median (IQR)	4 (4–5)	3 (2–8)	0.180
Days required to stop the need of supplement oxygen, median (IQR)	8 (7–10)	5 (4–5)	0.001
Patients required ICU support, *n* (%)	5 (29.4)	2 (10)	0.005
Patients intubated on ventilator, *n* (%)	2 (11.8)	1 (5)	0.141
Length of hospital stay (day), median (IQR)	15 (9–18.5)	12 (10–14)	0.028
30-day mortality, *n* (%)	1 (5.9)	1 (5)	0.906

NLD = no loading dose; LD = loading dose; SpO_2_ = peripheral capillary oxygen saturation; RA = rheumatoid arthritis; IQR = interquartile range; ICU = intensive care unit; *n* = number; % = percentage.

## 4 Discussion

This study found that a single 8 mg oral loading dose of baricitinib added to its daily 4 mg maintenance dose for up to 2 weeks exhibited better clinical outcomes in patients with moderate-to-severe COVID-19 than 4 mg daily oral dose regimen without having a loading dose. The targeted SpO_2_ (≥95%) was gained earlier in patients who received an early 8 mg of loading dose of baricitinib than the patients treated without a loading dose of baricitinib. Similarly, the requirement of supplement oxygen support was significantly reduced earlier in patients treated with an extra 8 mg of loading dose of baricitinib that the patients received only 4 mg daily maintenance dose.

A recent study showed that around 80% of patients with COVID-19 develop acute lung inflammation due to massive cytokine storm [3,5,6,7] resulting in hypoxemia, impaired hypoxic pulmonary vasoconstriction, and high altitude pulmonary edema leading to ARDS [3,8,17], which may result in death in 2–7% of patients with COVID-19 pneumonia [18]. Janus kinases, a tyrosine kinase, play its major anti-inflammatory role in the cytokine signaling pathways by constitutively binding to cytokine receptors. To potentiate a cytokine storm, proinflammatory cytokines need to transmit more signals through signaling pathways. In-role, more than 40 different types of cytokines transmit signals through JAKs, including JAK1, JAK2, JAK3, and tyrosine kinase-2 (TyK2) [13,18]. Baricitinib has an oral bioavailability of approximately 79%, plasma protein binding ability up to 50%, mean half-life of approximately 12.5 h (in RA), and shows serum drug level of approximately 100–300 nM following a 4 mg oral dose [13,19]. The low molecular weight baricitinib concentration-dependently inhibits JAK1 and JAK2 with high target specificity [13].

In addition, baricitinib suppresses the production of Type-I interferons (IFNs) from plasmacytoid dendritic cells (pDCs), inhibits the synthesis of interleukin (IL)-6 from B cells [20], and possesses strong anti-viral property by inhibiting endocytosis [21]. Therefore, down-regulation of signal transmission of proinflammatory cytokines through JAKs, and suppression of other intrinsic inflammatory pathways makes baricitinib a suitable anti-inflammatory drug therapy in the treatment of COVID-19 pneumonia. The additional strong anti-viral property of baricitinib along with its selective anti-inflammatory ability has attributed its superiority to other oral investigational anti-inflammatory drugs in the treatment of COVID-19 pneumonia.

The plasma drug concentration of baricitinib at 2–4 mg daily oral dose is sufficient to exhibit its anti-inflammatory role (JAKs inhibition) in RA [11,12], but, a standard dose of baricitinib to achieve its optimum therapeutic outcome in COVID-19 pneumonia is still under investigation. In a recent study with a small sample size showed an improved clinical outcome of patients with COVID-19 with baricitinib at 4 mg per day of oral dose for 2 weeks [14]. In this study, a 2-fold higher (2 × 4 mg) single loading dose of baricitinib followed by 4 mg daily dose showed better therapeutic response in the management of moderate-to-severe COVID-19 pneumonia, and a superior clinical outcome was attributed in patients (case group) within 2 weeks of therapy with reduced hospitalization time and mortality rate. The major limitation of this study was small study sample size, short duration of the study, no proven justification of using 8 mg loading dose of baricitinib, and unavailability of serum cytokines monitoring facility in the study setup.

## 5 Conclusion

Severe pneumonia associated with COVID-19 is a major cause of mortality in COVID-19 infection. No anti-inflammatory drug, including baricitinib for the treatment of COVID-19 pneumonia has yet been recommended. In this study, 2-week-long 4 mg once daily oral maintenance therapy of baricitinib following a single 8 mg loading dose in moderate-to-severe COVID-19 pneumonia showed faster return to normal respiratory function with reduced requirement of ICU and ventilator support, length of hospital stay, and mortality rate than a loading dose less than 4 mg once daily oral dose of baricitinib.
